This article has been retracted.

# Improved RRT-Based Moving Path Planning Algorithm for Teaching Reform and Innovation in Western Orchestral Ensemble Classes in Colleges and Universities

**DOI:** 10.1155/2022/4273761

**Published:** 2022-09-24

**Authors:** Wang Zhang

**Affiliations:** Music School of Liaoning Normal University, Dalian 100629, China

## Abstract

Western orchestral instruments in colleges and universities, as important instruments, occupy a central place in many bachelor's degree programs in music education. Music teaching reform and innovation are central to the creative wisdom of music teachers, their musical upbringing, and the lived experience of their students. For teachers, the process of pedagogical reform and innovation is the process by which teachers realize their own pedagogical ideals. Teachers must first be motivated; in the absence of motivation, any advanced teaching methods will become pale in comparison and lose their value and usefulness. Therefore, the construction of teaching activities requires teachers to take responsibility for the education and support of students, to align their teaching goals with the development of each student, to make the students' feelings closely connected to them, and to make them feel their value in the learning process. Starting from teaching western orchestral instrument ensembles in colleges and universities, this thesis uses the research method of improving RRT's moving path planning algorithm to explain and analyze some problems that arise in teaching western orchestral instrument ensembles in colleges and universities and puts forward constructive suggestions and recommendations.

## 1. Introduction

With the development of China's economy and the flourishing of various enterprises, China has more and more musical exchanges with countries all over the world, enabling China to accept more and more Western musical instruments and musical cultures. With the development of the times, Western musical instruments are becoming more and more popular in China. Many people are beginning to understand and learn musical instruments, and professional students are increasingly learning them. However, different instruments have different timbres and difficulties, so learners carefully study their choices. When studying Western music courses in our universities, we find that almost all of them are “one-way.” In the study of Western wind instruments, many students study flute and clarinet, but very few students study oboe and bassoon. In the study of Western wind instruments, many choose the cello and violin, significantly more than those who choose the viola. These events clearly indicate a serious imbalance in the scientific study of Western orchestral instruments in colleges and universities. With the booming development of Western orchestral music education in China's colleges and universities, there are college Western orchestral music professionals in higher music institutions [1]. After decades of efforts, the teaching of Western orchestral instruments in colleges and universities have entered a new stage of development. As an important instrument, the college Western orchestral instrument occupies a central place in many music education bachelor's degree programs. As students of Western orchestral instruments in colleges and universities, they should systematically master the basic knowledge of Western orchestral instruments in colleges and universities and know the laws of music education. At the same time, students may choose to teach orchestral music, chamber music, and choreography in the performing arts of music. While studying Western orchestral instruments, China needs to learn from its study abroad experience in certain areas. The most important approach in choreography programs in foreign schools is to encourage students to adopt a free-form learning model, as well as to encourage them to develop creative and inventive thinking as they understand and play music differently than they initially create it. Overseas schools often organize small recitals at school to allow students to identify and correct performance deficiencies based on their actual academic performance. At the same time, university student competitions are organized in foreign conservatories, and this type of competition can be called a campus singer competition. The purpose is to find new stars in orchestral performance and singing, to strengthen professional exchanges between universities, and to drive the development of universities. According to the situation abroad, the Western orchestral ensembles in our universities should adhere to the principle of freedom, according to the individual wishes of each student, and maximize the students' motivation so that they can organize more friendly games, including intercampus competitions and provide students with more opportunities for activities. Schools should try to encourage students to participate in song competitions held at home and abroad. Regardless of the results of the competitions, hammering and exercising are of utmost importance to the students. Since the music curriculum reform, the new curriculum has been designed and piloted for nearly a decade and subsequently implemented in several pilot provinces across the country. In recent years, the music curriculum reform has been carried out under the overall curriculum reform. Today, the largest basic education reform since the new Chinese education has entered the stage of practical implementation and adaptation. By thinking rationally about and grasping the curriculum reform process, the pace can be further adjusted and forged ahead. Knowing how to implement the curriculum reform is a question that every teacher involved in the curriculum reform must seriously think about. The reform and innovation of the teaching of Western orchestral ensembles in higher education is also a necessary step to meet the requirements of the time and society [2].

This thesis corresponds to the topic of “Music Teaching in Higher Education.” Starting from the teaching of Western orchestral ensembles in colleges and universities, this thesis explains and analyzes some problems in the teaching of Western orchestral ensembles in colleges and universities by using the research method of improving the RRT's moving path planning algorithm and puts forward constructive suggestions and recommendations. It is hoped that research and exploration of contemporary musical concepts and modes of upbringing in developed countries, as well as research and exploration of existing teaching models and teaching methods, will make useful and pioneering attempts to bring the overall teaching of Western orchestral ensembles in colleges and universities in China closer to the world trend. Finally, in the teaching and learning of the basic skills in Western orchestral ensembles, the teaching and pedagogy of the basic knowledge of Western orchestral ensemble classes, as well as the elaboration of the inner logic, should be taken into account in the core professional courses in related disciplines such as orchestra, chamber music, and choreography. Learning requires consideration of teacher specificity in the curriculum and special attention to the professional skills of the learner. It is hoped that the exploration of the subject of Western orchestral ensemble in colleges and universities will improve the updating of music pedagogy in Western orchestral ensemble in colleges and universities, the continuous mastery of teaching contents and teaching methods and the cultivation of more highly qualified Western orchestral ensemble students.

## 2. Research Background

As the cradle of musical talents and the place of musical and cultural exchange, universities have a special role in the development of Chinese music in the West. The teaching of Western orchestral instruments in colleges and universities is both a need for the development of Western music in China and the need for higher art to enter the campus and improve the quality of campus culture, as well as the need for students' era and spiritual struggle. Teachers should view the learning process of instrument composition as a dynamic process that enables teachers and students to learn more deeply from each other. The curriculum for Western orchestral instruments in higher education takes place primarily in the classroom. It is neither a one-way linear influence of the teacher on the students nor a one-way linear influence between the students, but an interaction between the teacher and the students [3]. In particular, music teaching and learning can develop healthily through the constant dynamic interaction between teachers and students in the classroom. Some universities do not have educational institutions that support Western orchestras. Some music teachers of Western orchestral instruments in colleges and universities teach simple methodologies, mainly music and performance, while neglecting the aesthetic skills of their students. The following problems currently occur in Western orchestral ensembles in our colleges and universities: training is inconsistent, the purpose of sound testing is to make each instrument sound almost identical, and rehearsals for musical integrity, unity, and completeness can be better accomplished at the same pitch. The relative instability of intonation still exists in the daily training and rehearsals of the orchestra. In daily orchestra practice and rehearsal, there are often differences between the beginning and the end of the piece. In daily orchestral practice, as the number and complexity of musical performances increases, the potential for complex rhythms, types, or sound types increases. Confronted with multisyllabic patterns, students can become ambivalent, fearful, or even too much bad, so practice is not reinforced. As part of the orchestra's daily curriculum, students need to be familiar with the music, and students are not guaranteed to play at a speed that can be reasonably controlled. Therefore, teachers in universities should currently pay attention to the teaching of music composition courses to develop students' musical aesthetic skills and thus improve their musical abilities [4]. Therefore, this thesis on the reform and innovation of teaching western orchestral instrument ensemble class in colleges and universities based on improved RRT's moving path planning algorithm has the following significance and principle requirements.

1. In the process of building vocal complexes in colleges and universities, teachers should strictly follow the three principles of subjectivity. The teaching of the Western orchestral instrument course in colleges and universities should fully reflect the dominant position of the students in the classroom. Teachers should change the traditional teaching attitude and fully stimulate students to learn practical skills in the teaching course of the Western orchestral instrument in colleges and universities. When constructing the Western orchestral instruments curriculum in colleges and universities, it is important to reflect on the joint harmony between teachers and students and to create a classroom environment where teachers and students have equal status. Teaching in higher education based on orchestras not only stimulates students' personal feelings but also forms their musical taste and aesthetic ability for music. Due to the influence of musical aesthetics on students' personalities, the teaching of the Western orchestral instruments in colleges and universities is receiving more and more attention from teachers [5].
2. Teachers in current university music teaching need to individualize instrumental-vocal instruction according to students' practical skills and choose appropriate teaching modes to arouse students' interest and motivation in music. In addition, interactive teaching can create a good environment for students to learn music and use music culture to learn music more deeply. In the teaching process, teachers should actively use multimedia to assist students in creating an open environment for teaching Western orchestral instruments in colleges and universities, so that they can focus more on cooperative lessons and take into account the teaching atmosphere created by teachers in the classroom to enrich the ensemble teaching content. Teachers in colleges and universities should not only have professional theoretical knowledge but also have a lot of practical skills. In the context of reforming the curriculum of Western orchestral instruments in colleges and universities, college teachers must break the traditional teaching model, develop new teaching concepts, and dare to use all innovative elements to change the existing curriculum of Western orchestral instruments [6].

## 3. Research Methods and Materials

### 3.1. RRT's Moving Path Planning Algorithm

#### 3.1.1. RRT Algorithm Concept and Formula

For the RRT algorithm, it is particularly important to define each expansion step of the moving path planning; if there is no synchronization, then the long time scheduling depends on time and cost. The computation of RRT is terminated when the random tree is expanded with new nodes [7]. The equation is as follows:

(1) $$\begin{array}{c} \mu_{X}=\mu_{M}+\frac{△x\left(\mu_{N}-\mu_{M}\right)}{\left\|\left(\mu_{N}-\mu_{M}\right)\right\|}\text{,} \end{array}$$

where △*x*, *μ*_*N*_ − *μ*_*M*_, and ‖(*μ*_*N*_ − *μ*_*M*_)‖ denote the random tree step size, vector unitization and Euclidean distance, respectively.

Delta-X expansion is a given value which has an important effect on the range of the random tree. If the extension length is small and the tree has many short branches, the path expansion speed can be effectively increased. However, from the beginning to the end, the random tree needs to be expanded step by step, requiring more nodes to find the workspace and find the solution, which reduces the efficiency. However, if the step size is larger, the random tree may have more branches, which will help to reduce the number of nodes required for the path. However, if there are too many obstacles in the room to complete the route planning, a large number of samples are required to obtain the extended nodes. This leads to path degradation too high, resulting in local extremes and even failure to find feasible paths [8]. The RRT algorithm flow is shown in Figure 1 and the RRT algorithm expansion schematic is shown in Figure 2.

#### 3.1.2. Advantages and Disadvantages of the RRT Algorithm

The main advantages of the RRT algorithm are as follows:

1. RRT algorithm is possible, i.e., it can be found if there exists a path from the start to the destination and the algorithm runs long enough [9].
2. The RRT algorithm can detect and evaluate obstacles in real time without the need to build a preconfigured spatial model.
3. The RRT algorithm is efficient and can even meet the requirements of real-time scheduling.
4. The RRT algorithm still has good performance in high-dimensional space, and it is relatively easy to extend the RRT algorithm from low to high dimensions [10].
5. The RRT algorithm is well adapted to dynamic environments. Even if the map information changes, it does not affect its effectiveness.

The main disadvantages of the RRT algorithm are as follows:

1. The study of the RRT algorithm is absolutely random. The RRT algorithm undergoes many invalid studies before an acceptable solution is found, which is an important factor affecting the effectiveness of the RRT algorithm.
2. The path generated by the RRT algorithm is not guaranteed to be the best solution, which is unlikely to be the optimal solution.
3. Even under the same laboratory conditions, the RRT algorithm is still unstable, which sometimes causes the RRT algorithm to fall into local minima.
4. The RRT algorithm must compare the distance between random nodes and extended nodes to determine the location of new nodes, which makes its computational efficiency gradually decrease as the number of nodes increases. Detection at this point has a high probability of redundancy.
5. In complex conditions such as narrow environments, most RRT calculations are used for obstacle detection, and the overall efficiency of the algorithm will be greatly reduced [11].

A comparison of the advantages and disadvantages of the RRT algorithm is shown in Figure 3.

#### 3.1.3. Path Planning

The route planning process involves obtaining information about the working environment through sensors and reliably determining the best transition path from the starting position to the target position in the working environment based on defined evaluation criteria (e.g., minimum energy consumption, shortest path, and shortest working time) [12]. The path planning equation is as follows.

(2) $$\begin{array}{c} l=\min\;\left\{\left.f\left(\delta \right)↔S_{n},\delta \in \left[0,1\right.\right)\right\}\text{,} \end{array}$$

where *l* equation represents the optimal path *f*(*δ*)↔*S*_*n*_.

### 3.2. Reform and Innovation of Music Teaching in Colleges and Universities

#### 3.2.1. Concept Update

In the past, music teachers in China's higher education institutions only focused on the teaching of music knowledge and skills, while neglecting the cultivation of students' practical and application skills. As a result, students' own knowledge and skills often cannot meet the needs of market development. Due to the influence of traditional teaching concepts, music language teachers also ignore students' subjective initiative in the teaching process and the passive learning process affects its effectiveness. To improve the quality of music teaching in colleges and universities, music teachers must carry out reform and innovation in the teaching process and pay due attention to students' initiative in the practical teaching process. They should fully and effectively stimulate students' interest in learning and more active participation in music teaching. Especially in a changing society, college music teachers must change their teaching attitude and clarify the main position of the class to ensure that students can create a more harmonious classroom atmosphere and improve their musical quality [13].

#### 3.2.2. Innovation of Methods

The current traditional music teaching methods do not adapt to the era of rapid economic development. The real needs of our market have limited the development of students. Therefore, it is necessary to reform and update the music teaching methods at this stage. On the one hand, music teachers in colleges and universities should deeply analyze the actual situation and personality characteristics of students in the teaching process, enhance the teaching relevance on the basis of reasonable selection of teaching contents and methods and effectively improve the students' music level. Music, as a unique art form, often puts higher demands on students' practical skills and creative ability. In both cases, teachers should also pay attention to developing students' abilities. At the same time, reform and innovation in teaching methods require teachers to change traditional assessment methods and apply more diverse approaches to improve overall assessment [14].

#### 3.2.3. Improvement of Music Teaching Institutions

The improvement of music teaching institutions is the basis for ensuring the quality of music teaching, so the reform and innovation of music teaching in colleges and universities must be promoted. At present, with the increase of the number of students in higher education institutions, the existing number of music education institutions in China's colleges and universities have not matched the existing number of students, which to a certain extent restricts the quality of music teaching in colleges and universities. Music teaching equipment, as the most important material guarantee for music teaching, not only plays a supporting role for music teaching but also directly affects its effect. In order to effectively improve the quality and level of their music, students need to use their free time outside of class, which usually requires schools to have adequate practice machines. Therefore, our universities need additional funds to improve the equipment and facilities for music teaching [15].

#### 3.2.4. Improvement of Professional Quality and Expertise

The professional quality and professionalism of music teachers in higher education often directly affect the quality of music teaching. Therefore, the reform and innovation of music teaching in colleges and universities also need the optimization and improvement of teachers' team. First of all, in recent years, the number of students in China's universities has been increasing, and the current number of teaching staff cannot meet the needs of the increasing number of students, which not only brings certain pressure to music teachers but also to the overall quality of music teaching. On this basis, our universities should focus on reforming and innovating music teaching, increasing the number of music teachers in schools and ensuring the comprehensive quality of music educators through strict enrollment; in order to improve the teachers' music teaching, our universities should also focus on strengthening the existing education and training of music teachers, improving their professional quality and level, and fundamentally improving their music education [16].

## 4. Results and Discussion

### 4.1. Experimental Discussion

In this part, the analysis of the Western orchestral instrument ensemble in China's colleges and universities using the improved RRT's moving path planning algorithm is mainly as follows.

1. The number of professional learners of the Western orchestral instrument ensemble in China's colleges and universities.
2. According to the data analysis, it can be seen that the number of people studying the Western orchestral instrument ensemble in China's colleges and universities from 2014 to 2022 has been increasing, mainly because the Western musical instruments are becoming more and more popular in China with the development of the time. Many people are beginning to understand and learn musical instruments and more and more professional students are learning musical instruments, as shown in Figure 4.
3. Teachers' participation in the teaching of Western orchestral ensemble in China's colleges and universities.
4. Assuming that the teachers' participation in the teaching of Western orchestral ensemble in China's colleges and universities is 100 points, the analysis of the data shows that the teachers' participation in the teaching of Western orchestral ensemble in China's colleges and universities is above 90 points, which proves that the teachers' participation in the teaching of Western orchestral ensemble in colleges and universities are extremely high, which limits the students' motivation to some extent, as shown in Figure 5.
5. Students' initiative in the teaching of the Western orchestral instruments ensemble in Chinese colleges and universities.
6. Assuming that the initiative of students in the teaching of Western orchestral ensemble in China's colleges and universities is 100 points, the analysis of the data shows that the initiative of students in the teaching of Western orchestral ensemble in China's colleges and universities is above 70 points, and the students' initiative is not enough, as shown in Figure 6.
7. Relationship between students' initiative and teachers' participation in the teaching of Western orchestral ensemble in colleges and universities in China.
8. Assuming that students' initiative in the teaching of Western orchestral ensemble in China's colleges and universities is scored 100 out of 100, and the horizontal axis indicates the teacher's participation, it can be seen from the data analysis that students' learning initiative score is getting lower and lower when the teacher's participation is from 10% to 90%. The quality of teaching is as shown in Figure 7.
9. Satisfaction of teachers and students in the teaching of Western orchestral ensemble in Chinese schools.
10. Assuming that the satisfaction score of teachers and students in the teaching of Western orchestral ensemble in Chinese schools is 100, the data analysis shows that the satisfaction score of teachers is above 70, and the satisfaction score of students is above 80, which proves that teachers and students are not very satisfied with the teaching of Western orchestral ensemble, so it is necessary to reform and innovate the teaching system of the curriculum, as shown in Figure 8.

### 4.2. Analysis of Results

#### 4.2.1. Problems of the Western Orchestra Ensemble Courses in Colleges and Universities

Students are not very enthusiastic about Western orchestral ensembles in orchestras. Some university teachers do not understand the importance of the Western orchestra course for training students and some students do not know what professional qualities and skills should be possessed by the Western orchestra ensemble, which leads to a decrease in students' enthusiasm for learning the Western orchestra. For some university teachers, learning the Western orchestra ensembles is an ongoing process. As students become less motivated in the learning process, the learning process is interrupted, which eventually leads them to learn poorly in the orchestra and even affects their future careers.

Some university teachers who teach Western orchestral music not only teach practical training methods for Western orchestral music but also teach courses on instrumental collaboration theory and Western orchestras. However, most students are not interested in the theoretical knowledge of the Western orchestras. Some students have not received specialized and systematic teaching and training, and the Western orchestral ensembles lack intonation and rhythm. The lack of awareness of some teachers about the importance of combining theory and practice makes it difficult for some students to give full play to their own initiative and motivation in learning.

In the teaching of vocal instrumental ensemble courses in higher education, some teachers strive only to improve the professionalism and integrity of vocal instrumental ensemble courses, which require different voices to achieve precise division, interaction and balance during performance. However, this requirement can only be achieved with the support of professional training, teamwork, and coordination skills. Any lapses in performance will directly affect the performance of the orchestra. However, some educational professionals in higher education institutions currently exhibit passivity or lack of professional cooperation, resulting in a somewhat unbalanced selection of the Western instruments, thus limiting the balance of string tone.

#### 4.2.2. Requirements for Western Orchestral Ensemble Courses in Colleges and Universities

*(1) Requirements for music teachers*. In practice, teachers should not only train students to play the instruments but also improve students' independent learning ability. This will enable students to develop good self-learning habits, to become familiar with the music independently before the lesson, to become familiar with the background of the music composition, and to understand the inspiration and meaning of the song composition. The students are taught according to their level of suitability. Different students' perception and understanding of music varies greatly; therefore, their ability to learn the Western orchestral instruments varies as well. In recent years, there has been a wide gap in the level of professional training of string students. These differences do not require teachers to generalize in practice, but rather to reinforce what students already know based on their level of learning. This requires teachers to design different courses and programs for each student. We develop different internship opportunities for different students. For students who have a good professional foundation and lack of practical work, teachers should find more opportunities for them to perform onstage and provide more opportunities for students to perform onstage. This will not only improve students' professionalism but also their adaptability and practical experience. In addition, these students can be encouraged to perform in house concerts, interact with students from other schools, and participate in music competitions. For students with a weak foundation, teachers should encourage them to improve their skills. Teachers will arrange appropriate music and music courses for these students, require them to take specialized subjects carefully when needed and ensure that they do not take exams. Students will be allowed to review the songs carefully after class and play them according to their understanding, giving them new life and meaning. We focus on a comprehensive curriculum. In terms of specialized courses, we should also schedule appropriate orchestra orientation courses. In orchestra orientation classes, students can simulate in the environment and train their reactions to the stage in a playful atmosphere [17].

Teachers need to pay more attention to changes in higher education policy and to the study of Western orchestras. Higher education teachers need to put themselves at the center of their learning, actively learn some theoretical knowledge related to the Western orchestral ensemble courses, and actively participate in artistic practices in and out of school. The traditional method of cooperative learning is reading and games. They neglect choral lessons like other subjects, which cannot be understood solely through collegial learning. Teachers can make full use of multimedia technology for reading, teaching, presenting, and teaching. While playing the Western orchestral instruments, the teacher must take the lead in rehearsing, cooperating, and working closely together in order to play beautiful music under the guidance of the conductor. Therefore, it is necessary to coordinate theoretical teaching, integrate professional masters and teachers, equip students with the ability to combine conducting and performance, and integrate the teaching resources of the Western orchestras. In schools that are in a position to attract all relevant professional teachers to form an orchestra, professional teachers can specifically train each voice of the student orchestra in order to improve the students' professionalism within the orchestra and facilitate the integration of the orchestra into the performance process. For some students, it is easy to become distracted and interested in something new in the classroom. Considering the psychological development of the Western orchestra students at this stage, during this time, teachers can recreate instruments, such as string, wind, and other components, and can use the unique sonic characteristics of these instruments to foster active exploration and creative thinking as students learn the instruments. Students are allowed to choose their own notes or substitute original instruments. In addition, as part of teaching western orchestral ensembles, teachers should make full use of various teaching materials and design individualized teaching forms and methods to make teaching Western orchestral ensembles richer and more interesting, thus stimulating students' interest in music more effectively. Teaching Western philharmonic music is an integral part of music teaching in higher education. Accurate rhythm and intonation are the keys to good music. Teachers should understand the difficulties of teaching college orchestras, think deeply about sound teaching methods, apply interdisciplinary, fixed-pitch models to support sound teaching, strengthen students' foresight, and help them develop a sense of proper high level. Teaching evaluation is highly abstract, but most students have a weak sense of abstraction, and disqualification theory often underestimates the meaning and emotional understanding of the work, most often by listening to the music. Combining teaching with comprehension not only allows students to feel the melody of the music more realistically but also reflects the resonance of ideas and emotions, as if they were in the real world, feeling the power of music [18].

*(2) Requirements for students*. Students are at a stage where they are interested in new subjects. Teachers should take full advantage of these qualities of their students to develop more relevant teaching methods. In Western orchestra instruction, students can only remember the specific rhythms of the notes, not the unique art of the notes. However, if classroom teachers use multimedia technology to represent rhythm in three dimensions in musical performance, they can provide students with a visual and audio-visual three-dimensional musical composition that immerses them in musical appreciation. In evaluating this form of music, students form images and perceptions that are consistent with the notes and have the pedagogical and cognitive potential to enable them to understand the notes in greater depth. Therefore, in the current collaborative teaching, teachers should actively introduce multimedia technology in collaborative teaching so that students can improve their music perception and music perception skills in the learning process [19].

For university teachers, more effective and comprehensive development is inseparable from the university teaching environment and teaching resources. Universities have reformed their teachers at the request of professional associations of education, changing the curriculum of the Western orchestra, and making innovations. The University hires professional faculty members to provide more effective professional advice to young faculty members of higher education institutions, to provide more teaching resources to students, to provide a good learning environment so that they can better develop their acting skills and develop their abilities to express their emotions through instrumental orchestral works, to enable students to combine the theory and practice of the Western orchestra, and to develop their comprehensive skills in order to meet their professional qualities and the higher education in social sphere. In teaching the Western orchestras, teachers should introduce students to the personal emotions that Western music conveys in the teaching process in order to reduce students' tension in collaborative teaching. At the same time, the musical function helps students to establish independent learning patterns. In the teaching process of western orchestral ensembles, teachers can combine the original musical features through interaction and collectivism to encourage students to create their own compositions in daily teaching, so that students can give full play to their creativity and imagination in the sea of music. At the same time, teachers can assess students' creative notes according to their individual characteristics, actively provide tutoring and targeted teaching, and improve students' ability to acquire knowledge and appreciate music. Teacher-student collaboration is an effective way to teach university orchestras. Schools can hire world-class professional artists to serve as sound engineers for the Western orchestras, and students can have them play their instruments, ensuring both the stability and the sonic balance of the core members of the orchestra. However, one will also learn many of the benefits of professional musicians from them, helping the orchestra grow together. In addition, the formation of the strings needs to be relatively stable. It is not enough to rely on students alone, as they are more mobile. After a few years of training, they are just maturing, but they have to leave the orchestra because they are about to graduate. That is why the orchestra is like a cast iron camp and the sailors are like a cycle, one after the other. The people in the orchestra change every year and every year people leave the orchestra. The orchestra was founded in the most difficult period of development, in the middle of a small water period. To solve this problem, professional teachers are required to participate in orchestra rehearsals, and each mainstream music school needs the support of one or two teachers to maintain relative stability [20].

## 5. Conclusion

With the rapid development of the political and economic life of the country, the level of musical, cultural, and artistic activities of the society is also increasing. According to the demand of the society for musical talents, it is the primary task of the higher music majors to cultivate musical and artistic talents suitable for Chinese conditions. However, the Western orchestral instrument courses in higher education institutions are still in the primary stage. Educational philosophy, training objectives, curriculum design, and teaching methods are usually organized according to the pattern of general higher education. The lack of professional experience of teachers, the weakness of students' professional foundation, the lack of understanding of the concept of “qualification standards” in higher education, the lack of “functional and innovative” training, and the development of the Western orchestral instruments in higher education are limited by a number of factors, such as the lack of acceptance of social and professional needs and the lack of talent. The development of the Western orchestral instruments in universities is limited by a number of factors, such as the lack of acceptance of social and professional needs, the characteristics of human resources training, and differences in professional positions. From a macro perspective, this thesis explains and analyzes some problems in the teaching of Western orchestral ensembles in colleges and universities from a practical point of view and puts forward constructive suggestions and recommendations by using the research method of improving RRT's moving path planning algorithm. The reform of talent model in higher music institutions should adapt to the demand of society for music teachers and talents in the new era and to the new changes in the field of basic education reform and basic education. However, considering the new requirements of the new era, the reform of music education in higher music institutions lacks effective means. The reform must be a long-term process, requiring continuous research and experimentation. Therefore, music study programs should be modified and adapted to accommodate the transformations required by the new era in order to produce musicians who may be useful to society. The reform of higher music education should focus on how to maintain the strengths of teaching music skills and fill the gaps in practical courses such as teacher training. Music education should be oriented to the needs of society and clearly oriented to the educational objectives, and in the teaching system, it should be oriented to the training model of music teachers. The concept is based on the talent development model, and the system construction and teaching management should be strengthened to ensure the talent development model. Of course, the road of reform is not smooth, but it will also encounter resistance. The main force of music education professional reform is the first year teachers. They should pay more attention to teaching research. Teachers can only be a permanent source of strength to implement class reforms and to carry out reform measures if they reach a consensus. Unlike general higher education, the goal of higher education talent training is closely related to the social occupation or professional process. Higher music education should go out of the standard basis of music specialization in general higher education system, boldly reform, constantly innovate, fully consider the needs of social music profession, take professional development as the guide, take employment as the guide, clarify the university music career goals, form curriculum model and system, establish corresponding teaching talents and diversified evaluation mechanism, fully reveal the value of music talents, highlight the characteristics of higher education, and improve the social competitiveness of musicians, train musicians, and meet the needs of society. Through studying the Western orchestral ensembles, we have gained a deeper understanding of the Western orchestral instruments. As a cradle of musical talents and a place of musical and cultural exchange, universities have a special role in the development of Chinese music in the West. The teaching of the Western orchestral instruments in colleges and universities is both a need for the development of the Western music in China and a need for higher arts to enter the campus and enhance the cultural quality of the campus, as well as a need for the students' age and spiritual struggle. Given the current situation in China, we must do more to implement effective curriculum reform and development. In terms of training programs, in addition to the basic professional courses, relevant courses such as chorus, band section leadership, and orchestra rehearsal should also be added. We should make the curriculum innovative, based on previous knowledge, more interesting and professional so that students can gain more knowledge and experience in a more favorable environment. It is also worth thinking about the fact that the musicianship courses for the Western orchestral instruments in our universities provide students with good theoretical training and practical orchestral skills, making them more powerful and socially competitive in the future work process.

## Figures and Tables

**Figure 1:** RRT algorithm flow.

**Figure 2:** RRT algorithm expansion schematic diagram.

**Figure 3:** Comparison of advantages and disadvantages of the RRT algorithm.

**Figure 4:** Number of professional learners of the Western orchestral instruments ensemble in China's colleges and universities in the recent years.

**Figure 5:** Teacher involvement in the teaching of the Western orchestral instrument ensemble in colleges and universities in China.

**Figure 6:** Students' initiative in the teaching of the Western orchestral instrument ensembles in colleges and universities in China.

**Figure 7:** Relationship between students' initiative and teachers' involvement in teaching Western orchestral ensemble in Chinese universities.

**Figure 8:** Satisfaction of teachers and students in the teaching of the Western orchestral instrument ensemble in our school.

## Data Availability

The dataset is available upon request.
